The article "The role and molecular mechanism of Trop2 induced epithelial‐mesenchymal transition through mediated β‐catenin in gastric cancer" was retracted in 2025. Reasons: manipulated data; manipulated images; duplicated images; duplicated data.

# The role and molecular mechanism of Trop2 induced epithelial‐mesenchymal transition through mediated β‐catenin in gastric cancer

**DOI:** 10.1002/cam4.1934

**Published:** 2019-01-11

**Authors:** Wei Zhao, Lizhou Jia, Xingwang kuai, Qi Tang, Xiaochen Huang, Tingting Yang, Zhenning Qiu, Jin Zhu, Jianfei Huang, Wenbin Huang, Zhenqing Feng

**Affiliations:** ^1^ Department of Pathology, Nanjing First Hospital Nanjing Medical University Nanjing China; ^2^ Department of Pathology Nanjing Medical University Nanjing China; ^3^ Key Laboratory of Antibody Technique of Ministry of Health Nanjing Medical University Nanjing China; ^4^ Huadong Medical Institute of Biotechniques Nanjing China; ^5^ Department of Pathology Affiliated Hospital of Nantong University Nantong China; ^6^ Jiangsu Key Lab. of Cancer Biomarkers, Prevention and Treatment, Collaborative Innovation Center for Cancer Personalized Medicine Nanjing Medical University Nanjing China

**Keywords:** epithelial‐mesenchymal transition, gastric cancer, Trop2, β‐catenin

## Abstract

The present study elucidates the potential role of Trop2 in tumor invasion and the promotion of epithelial‐mesenchymal transition (EMT) when binding β‐catenin in GC. The role of Trop2 in promoting EMT in GC cells was examined by a variety of experimental assays. Moreover, the underlying molecular mechanism of Trop2 in promoting EMT was studied by in vivo and in vitro assays. The Trop2 expression in relation to tumor metastasis status was detected by IHC in 248 cases of GC tissues and 86 cases of matched adjacent tissues. Trop2 promoted the metastasis and induces EMT in GC. Meanwhile, the elevated protein levels of Trop2 and mesenchymal markers were also found in the TGF‐β1‐induced EMT model in GC cells. Importantly, Trop2 physically bound and activated β‐catenin to promote EMT; moreover, Trop2 increased the accumulation of β‐catenin in the nucleus to accelerate metastasis in GC cells. Inhibition of Trop2 expression in GC cells prevented the migration and invasion of GC cells in vivo. Trop2+/vimentin+ expression was higher in GC tissues than that in matched adjacent tissues, and Trop2+/vimentin+ expression in GC was associated with the differentiation, TNM stage, and distant metastases. These sets of data reveal a novel regulatory network of Trop2 in EMT and GC metastasis, suggesting Trop2 as a useful marker for inducing EMT and metastasis of GC, which may help to lead a better understanding of the pathogenesis of the GC.

## 1 INTRODUCTION

Gastric cancer (GC) is the most common digestive system malignancy and ranks as the third leading cause of cancer mortality worldwide.^1^, ^2^ Despite a declining rate of GC over the past decades,^3^ the 5‐year survival rate of GC patients is <20%.^4^ Moreover, no less than two‐thirds of GC occurs in developing countries, and China has the most GC patients in the world.^5^, ^6^ Despite significant medical progress and efforts in promoting the survival of GC patients, the basic molecular mechanisms of the GC are until recently still not well understood. Therefore, it is still important to identify novel diagnostic biomarkers and prognostic strategies.

Human trophoblast cell surface glycoprotein (TACSTD2/Trop2/M1S1/GA733‐1) gene is located at chromosome 1q32 and is a 36 amino acid transmembrane protein expressed primarily in epithelial cells.^7^ Trop2 first has been identified in human trophoblasts and has several binding partners, including claudin 1, 7, cyclin D1, protein kinase C (PKC), and PIP2.^8^, ^9^, ^10^ Trop2 can induce tight junctions at the epithelial barrier,^11^ and promote tumor proliferation, podosome formation, and the activation of Raf and NF‐kappa,^8^, ^11^ it can also inhibit IGF‐1R signaling by binding to these partners.^12^ Trop2 has been found over‐expressed in various epithelial tumors,^10^, ^13^, ^14^, ^15^, ^16^ and its expression relates to aggressive tumor behavior.^17^, ^18^

Epithelial‐mesenchymal transition (EMT) is a developmental process in which epithelial cells loss its phenotype and mesenchymal cells gain its phenotype, is considered to have an important role in the invasive and metastasis progression in the cancer.^19^, ^20^, ^21^ Moreover, EMT contributes to early‐stage metastasis and invasion of cancer cells.^22^ The process of EMT includes the decrease of epithelial markers such as E‐cadherin, mesenchymal, upregulation of markers, such as fibronectin, vimentin, and abnormal translocation of β‐catenin.^23^, ^24^ EMT processes have been reported to be initiated by zinc‐finger transcriptional repressors, such as snail or β‐catenin. Vimentin is known as one kind of mesenchymal marker, and upregulated vimentin is related to a poor clinical prognosis caused by many cancers including GC. But the underlying molecular mechanism of EMT processes still remains to be fully studied.

In 2014, Chen et al performed immunohistochemistry to observe the expression of Trop2 and EMT marker in gallbladder cancer. The results indicated that high Trop2 expression was significantly associated with lower E‐cadherin expression and acquisition of expression of vimentin.^25^ In our previous study, we also found Trop2+/E‐cadherin−was expressed in breast cancer (BC) and was associated with lymph node status, metastasis, tumor‐node‐metastasis (TNM) stage, and ER−/PR−/HER2− expression. Furthermore, BC patients that expressed Trop2+/E‐cadherin−had poor overall survival rates.^26^ But in these studies, the underlying molecular mechanism of Trop2 and EMT did not be fully studied.

In the present study, we found that Trop2 promoted EMT phenomenon and induced metastasis in GC. We further identified that Trop2 physically bound to β‐catenin and then increased mesenchymal markers as well as inhibited epithelial markers. Moreover, we also found that Trop2 promoted the nuclear accumulation of β‐catenin. Inhibition of Trop2 expression in GC cell lines inhibits migration and invasion both in vivo and in vitro*. *Finally, we identified that Trop2 expression positively correlated with tumor metastasis status in GC patients. Collectively, we identified potential invasion activities of Trop2 in GC cells, suggesting that Trop2 might be a promising therapeutic target for blocking the progression of GC.

## 2 METHODS

### 2.1 Tissue sample

A total of 330 formalin‐fixed, paraffin‐embedded (FFPE) stomach tissue samples, including cancer tissues (n = 248) and matched adjacent tissues (n = 86), were collected from 248 patients with primary GC who had undergone routine GC resection. All tissue blocks were received from the department of pathology at the Affiliated Hospital of Nantong University from 2003 to 2010. Tissue patients’ clinical medical records included age, gender, tumor‐node‐metastasis (TNM) stage, histological type, and differentiation grade. No patients received any treatment (chemotherapy, radiation therapy, or immunotherapy) before surgical resection. Overall survival (OS) was defined as the period from initial diagnosis via biopsy to death. Information on patients who were alive at the last follow‐up date was deleted from the analysis. The study protocol was approved by the Human Research Ethics Committees of the hospital.

### 2.2 Cell culture, reagents, and plasmid

Seven human GC cell lines (MKN45, MKN28, MGC803, MGC823, SGC7901, HGC27, and BGC823) and normal human gastric epithelial cell lines (GES‐1) were purchased from KeyGEN BioTECH (Nanjing, China). Cells were cultured in at 37°C in a 5% CO_2_ humidified atmosphere in RPMI‐1640 containing 10% FBS. Recombinant human TGF‐β1 was purchased from Novoprotein. The sequences for Trop2 overexpression vector and control OE vector, Trop2 shRNA and control shRNA vector are listed in Table S1.

### 2.3 RNA extraction, reverse transcription, and qRT‐PCR

Cell RNA was extracted by TRIzol reagent (Invitrogen, Carlsbad, CA, USA) and reverse transcribed into cDNA using a PrimeScript™ RT reagent kit (Takara, Glen Burnie, MD) in accordance with the manufacturer's instructions. The primers of Trop2 were β‐catenin, E‐cadherin, fibronectin, vimentin，goocecoid, and snail. GAPDH (internal control) was purchased from GENEray (shanghai, China). qRT‐PCR was performed on an ABIPRISM 7500HT Sequence Detection System (Applied Biosystems, Foster City, CA, USA) in 96‐well plates. Relative expression levels were calculated as ratios normalized against those of GAPDH. Results were normalized to respective internal controls. The Ct‐value for each sample was calculated using the ΔΔCt method, and results were expressed as 2^−ΔΔCt^. Primers can be found in Table S2.

### 2.4 Western blot analysis and co‐immunoprecipitation

Cellular proteins were lysed using standard methods. Cellular proteins were separated by 10% SDS‐PAGE and transferred onto nitrocellulose membranes. The membranes were blocked with TBS containing 0.1% Triton X‐100 and 5% nonfat milk for 2 hours at RT and then were incubated with Trop2 (R＆D SYSTEMS), E‐cadherin (Invitrogen), fibronectin (Affinity), vimentin (Affinity), β‐catenin (Santa Cruz Biotechnology), and β‐actin antibody (Abcam) at 4°C overnight. After being washed, the membranes were incubated with HRP‐conjugated anti‐IgG at RT for 1 hour. Signal detection was carried out with an ECL system (Tanon, shanghai, China). BGC823 and MGC803 were transfected with different plasmids and then lysed in cellular lysis buffer (Sangon Biotech, Shanghai, China) for 15 minutes on ice. Extracts were clarified by centrifugation at 13 000 *g* for 25 minutes at 4°C for co‐immunoprecipitation. After centrifugation, the supernatant was collected, and then incubated with protein G PLUS‐agarose immunoprecipitation beads (Santa Cruz Biotechnology) at 4°C for 1 hour. Then, they were incubated with special antibodies against Trop2, β‐catenin at 4°C on a rocker platform. The antibody‐coated beads were then incubated with the lysates at 4°C overnight. Immunoprecipitates were collected, washed, lysed, and boiled. The boiled samples were analyzed by Western blot analysis as describe above.

### 2.5 Immunohistochemical staining

The streptavidin‐peroxidase (SP) staining technique was used to detect protein following antigen retrieval by microwave treatment. After blocking endogenous peroxidase activity by incubating in 3% H_2_O_2_, tissues were placed in 0.01 mol/L citrate buffer, pH 6.0, and heated in a microwave for antigen retrieval. Trop2 was detected using a polyclonal goat anti‐human Trop2 (dilution 1:200), fibronectin (dilution 1:300), E‐cadherin (dilution 1:300), and vimentin (dilution 1:300). Antibody reactions were detected with an Envision™ peroxidase kit (Dako, Carpinteria, CA, USA). Tissues were then incubated in 3, 3ʹ‐diaminobenzidine plus (Dako), counterstained with hematoxylin, dehydrated through graded alcohols, and cleared in xylene. The following staining intensity scores were used: 0 indicated no staining; 1+ indicated weak staining; 2+ indicated moderate staining; and 3+ indicated intense staining. The total number of cells at each intensity level was multiplied by the corresponding intensity score to yield an intensity percentage score. Final staining scores were then calculated by summing the four intensity percentage scores; the minimum possible final staining score was 0 (no staining), and maximum possible score was 300 (100% of cells with 3+ staining intensity).

### 2.6 Migration and invasion assays

For transwell migration assays, transfected cells (4 × 10^5^) were plated in the top chamber with the non‐coated membrane (24‐well insert; pore size, 8 μm; BD Biosciences, San Jose, CA, USA). For invasion assays, matrigel (BD biosciences) was polymerized in transwell inserts for 2 hours at 37°C. In both assays, cells were plated in the top chamber in medium without serum; the lower chamber was filled with 10% FBS and EGF (25 ng/mL) (Sigma, St Louis, MO, USA). Cells were incubated for 24 hours, and the cells that did not migrate or invade through the pores were removed by a cotton swab. Cells on the lower surface of the membrane were stained with crystal violet and counted.

### 2.7 Cytoplasmic and nuclear extraction

Cytoplasmic and nuclear extraction lit for cells purchased from invent Biotechnologies. Inc The internal reference of nuclear protein was used with Lamin B1, and the internal reference of cytoplasmic was used with β‐actin. Harvest cells in suspension by low‐speed centrifugation and wash the cells through cold PBS. Collect the cells to a 1.5 mL‐microcentrifugation tube and centrifugate at 500 *g* for 1 minute, abandon supernatant, add appropriate amounts of cytoplasmic extraction buffer to cell pellets, vortex the tube vigorously, incubate on ice for 5 minutes. The procedures of cytoplasmic and nuclear protein extraction as descript in protocol.

### 2.8 Immunofluorescence assay

The inoculated trypsinized cells were placed in cell culture dishes (6 well) and incubated with vimentin antibody, fibronectin antibody, E‐cadherin antibody, Trop2 antibody, and β‐catenin antibody for 2 hours at room temperature, respectively, then incubated with fluorescent anti‐IgG at RT for 1 hour. A fluorescence microscope or confocal laser scanning microscope was used to detect the levels of the markers.

### 2.9 Animal experiments

Animal experiments were performed with the approval of the Institutional Committee for Animal Research and in conformity with national guidelines for the care and use of laboratory animals. ShRNA‐Trop2, shRNA‐NC‐infected BGC823 cells, and PBS were injected into the tail vein of immunodeficiency nude mice (n = 5). After 5 weeks, the mice were killed and metastatic lung tissues were used to analyze Trop2, fibronectin, E‐cadherin, vimentin protein expression.

### 2.10 Statistical analysis

The SPSS18.0 statistical software package (SPSS Inc, Chicago, IL) was used for general statistical analysis. The differences between groups were estimated by unpaired Student's *t *test. Overall survival (OS) rates were calculated by the Kaplan‐Meier method with the log‐rank test applied for comparison. Survival data were evaluated using univariate and multivariate Cox proportional hazards model. Values of *P *< 0.05 were considered statistically significant.

## 3 RESULTS

### 3.1 Trop2 induced metastasis through upregulated mesenchymal markers and downregulated epithelial markers

In our previous study, we detected the function of Trop2 in GC in vivo and in vitro. We found Trop2 to be an oncogene that can promote GC cell proliferation, apoptosis and induce G1‐S cell cycle progression in GC cell lines. But interestingly, our study also testified to the effect of OE‐Trop2 on cell migration and invasion. We analyzed the effect of shRNA‐Trop2 on cell migration and invasion. For shRNA‐Trop2 and shRNA‐NC (transfected MKN45 and BGC823 and then cultured in transwell apparatus), after 24 hours of incubation, the percentage of migrated cells in shRNA‐Trop2 transfected (two cell lines) were significantly lower than the shRNA‐NC cell group. By using a boyden chamber coated with matrigel, we determined that shRNA‐Trop2 could inhibit BGC823 and MKN45 cell invasion after being transfected for 48 hours (Figure 1A).

**Figure 1:** Trop2 induced metastasis through upregulated mesenchymal markers and downregulated epithelial markers. A, Trop2 knockdown inhibits metastasis in MKN45 and BGC823 by transwell migration assay and transwell invasion assay. The number of migrated and invaded cells was counted under the panel, respectively, mean ± SD, **P < 0.001, means compared with the shRNA‐NC control group. B, Overexpression of Trop2 prompts metastasis in MKN28 and MGC803 by transwell migration assay and transwell invasion assay. The number of migrated and invaded cells was counted under the panel, respectively, mean ± SD, **P < 0.001, means compared with the VE‐Trop2 control group. C, Representative Western blot results for fibronectin, E‐cadherin, vimentin, and Trop2 protein expression from OE‐Trop2 or shRNA‐Trop2 treated with MGC803 and BGC823 cell lines, GAPDH was used as a control. **P < 0.001, means compared with the NC control group. D, The mRNA level of mesenchymal markers and epithelial marker, expressed in OE‐Trop2 or shRNA‐Trop2 treated with GC cell lines, was analyzed by qRT‐PCR. GAPDH was used as a control. E, The mRNA level of EMT regulators (β‐catenin, goocecoid, snail), expressed in OE‐Trop2 or shRNA‐Trop2 treated with GC cell lines, was analyzed by qRT‐PCR, GAPDH was used as a control. All experiments were carried out in triplicate

For OE‐Trop2 and EV‐Trop2 plasmid (transfected MKN28 and MGC803 cultured in transwell apparatus), following 24 hours of incubation, the percentage of migrated cells in OE‐Trop2 transfected (in MGC803) were significantly higher than EV‐Trop2 group. Using a boyden chamber coated with matrigel, we found that OE‐Trop2 was able to increase cell invasion in MGC803 after transfected for 48 hours. But we did not observe a similar result in the MKN28 cell line (Figure 1B). It may be the reasons of lower transfection efficiency.

To evaluate whether Trop2 affects the EMT phenomenon in GC cells, we over‐expressed Trop2 in MGC803 and knockdown Trop2 expression in BGC823, then examined the expression of the epithelial marker (E‐cadherin) and mesenchymal markers (fibronectin and vimentin) by Western blot (Figure 1C) and qRT‐PCR (Figure 1D). Trop2 overexpression led to *increased* fibronectin and vimentin protein expression, but conversely decreased E‐cadherin protein expression. Then, with knockdown Trop2 (by shRNA‐5‐Trop2), the fibronectin and vimentin protein expression decreased and E‐cadherin protein expression increased. The mRNA profile was similar to the protein expression.

To detect which EMT regulators might be influenced by Trop2, we used qRT‐PCR to evaluate the expression level of several EMT regulators after applying OE‐Trop2 in MGC803 and shRNA‐Trop2 in BGC823. We found the expression level of β‐catenin and Trop2 was positively correlated (Figure 1E).

Collectively, this observation indicated that Trop2 might play an important role in regulating EMT phenomenon in GC cell lines.

### 3.2 Trop2 physically associated with β‐catenin to induce EMT phenomenon

To further elucidate whether Trop2 plays a role in the EMT regulation phenomenon, we used transforming growth factor β1 (TGF‐β1) to induce EMT regulation in GC cell lines (MGC803 and BGC823) (Figure 2A). After TGF‐β1 was stimulated for 7 days, we observed the morphological changes in the MGC803 and BGC823 gastric cancer cell lines by microscopy (magnification: 400). Meanwhile, we examined the epithelial and mesenchymal markers, and Trop2 protein expression of TGF‐β1 induced GC cell lines by fluorescence microscopy (Figure 2B) and qRT‐PCR (Figure 2C). We found that the fibronectin, vimentin, and Trop2 protein expression increased but E‐cadherin protein expression decreased.

**Figure 2:** Trop2 physically associated with β‐catenin to induced EMT phenomenon. A, TGF‐β1 induced morphologic changes in MGC803 and BGC823 GC cell lines by phase‐contrast microscopy (magnification: 400), fibronectin, E‐cadherin, vimentin, and Trop2 expressed in two types of GC cell lines or TGF‐β1‐treated GC cell lines by fluorescence microscopy (magnification: 400) (B) and qRT‐PCR(C). D, The change of the EMT regulators after TGF‐β1 induction by qRT‐PCR. E, Analysis of the interactions between Trop2 and β‐catenin using STRING database. F, MGC803 cell lysates were pre‐immunoprecipitated with anti‐Trop2 or anti‐β‐catenin antibody, and the co‐immunoprecipitated β‐catenin or Trop2 was detected using anti‐β‐catenin or anti‐Trop2 antibody, WCL means whole cell lysate, IC means immune complexes. G, Vimentin, Trop2, and β‐catenin protein expression level in EMT model cell lines and shRNA‐Trop2‐treated EMT model cell lines by Western blot, GAPDH was used as a control, mean ± SD, **means compared with NC group, *P* < 0.001. All experiments were carried out in triplicate

We examined the EMT regulators (β‐catenin, goocecoid and snail) in induced GC cell lines (EMT model cell lines) by qRT‐PCR (Figure 2D). The result indicated that the change of the β‐catenin in two EMT model cell lines, compared to normal GC cell lines, was more significant than others (EMT model cell line MGC803 vs normal MGC803: 3.88 ± 0.59, EMT model cell line BGC823 vs normal BGC823:2.72 ± 0.53). These results showed that EMT key regulator β‐catenin might target EMT markers for its transcription in GC. We carried out STRING database analysis (http://www.string-db.org/cgi/network.pl?taskId=CfBlxq0SyuCt) to analyze the interactions between the known proteins and the predicted proteins. The result indicated that Trop2 and β‐catenin in the cell junction and cell signaling pathways may have a certain role (Figure 2E). Therefore, we hypothesized the potential involvement of Trop2 and β‐catenin in the EMT phenomenon. To further characterize the correlation between Trop2 and β‐catenin, we performed a co‐immunoprecipitation experiment in the MGC803 cell lysates (immunoprecipitated with anti‐Trop2 antibody or anti‐β‐catenin). The co‐immunoprecipitated β‐catenin or Trop2 was detected using an anti‐β‐catenin antibody or Trop2 antibody, and the physical interaction of Trop2 with β‐catenin was observed (Figure 2F).

Next, we detected the changes in Trop2, β‐catenin, and vimentin protein expression in the GC cell lines, EMT model GC cell lines, shRNA‐NC EMT model GC cell lines, and shRNA‐5‐Trop2 EMT model GC cell lines, respectively. We found that TGF‐β1 could induce vimentin, Trop2, and β‐catenin protein expression in two GC cell lines (MGC803 and BGC823), whereas knockdown Trop2 in EMT model GC cell lines could downregulate vimentin and β‐catenin protein expression compared to the control group (Figure 2G). Furthermore, we witnessed the change of vimentin and β‐catenin protein expression in the overexpression or knockdown Trop2 of the MGC803 and BGC823 by immunofluorescence assay with confocal microscopy. The result indicated that OE‐Trop2 is able to induce a higher expression in vimentin and β‐catenin protein, whereas shRNA‐Trop2 show the ability to inhibit these protein expression levels (Figure 3A‐D). Then, we detected the vimentin and β‐catenin protein expression in Trop2 inhibition or TGF‐β1‐induced Trop2‐depleted BGC823/MGC803. We found that when OE‐Trop2 or TGF‐β1 was induced, it could promote β‐catenin nuclear accumulation and vimentin expression in the cell membrane, but shRNA‐Trop2 could *inhibit* expression in MGC803 and BGC823 (Figure 3E‐H). Thus, Trop2 is required for β‐catenin nuclear accumulation and induced mesenchymal markers expression during the EMT process in GC cell lines.

**Figure 3:** Trop2 positively mediated TGF‐β1‐induced β‐catenin nuclear accumulation by immunofluorescence assay with confocal microscopy (magnification: 400). Vimentin and β‐catenin expressed in MGC803 and OE‐Trop2‐MGC803 group (A and B), BGC823 and shRNA‐Trop2‐BGC823 (C and D). Detected vimentin and β‐catenin expression level of the shRNA‐NC, TGF‐β1 + shRNA‐NC, and TGF‐β1 + shRNA‐Trop2 treated with two types of GC cell lines(E‐H). I, The expression level of β‐catenin in nucleus and cytosol in OE or shRNA‐Trop2 GC cell lines, Lamin B1 as a control in nucleus, β‐actin as a control in cytosol. Mean ± SD, **means compared with NC group, *P* < 0.001 (I). All experiments were carried out in triplicate

To further detect the relationship of Trop2 and β‐catenin in GC cells, we performed separation technology of nucleus and cytosol. The results indicated that OE‐Trop2 in MGC803 could induce the expression level of β‐catenin in cell nulear, while inhibit that in cell cytosol. And then, shRNA‐Trop2 in BGC823 have the adverse results (Figure 3I).

### 3.3 Trop2 depletion inhibits metastasis of GC cell line in vivo

To assess the effects of shRNA‐Trop2 on the metastasis of the GC cells in vivo, we constructed a tail vein injection transfer model. shRNA‐Trop2 and shRNA‐NC plasmid‐transfected BGC823 cells (1 × 10^6 ^cells/mouse) were injected into immunodeficient nude mice tail veins (n = 5/group), then compared with the PBS injected into the tail vein of the control group mice (n = 5/group). After 30 days, the mice were sacrificed, and then, their lungs were examined. The lungs from the mice injected with shRNA‐NC and shRNA‐Trop2 treated with BGC823 cells were larger and heavier than those from PBS control group, and those from shRNA‐NC group were larger and heavier than those from shRNA‐Trop2 group (*P* < 0.05; Figure 4A). In a representative picture of lungs from shRNA‐NC group and shRNA‐Trop2 group, we detected some micrometastasis (Figure 4B), moreover, the number of tumor colonies in shRNA‐NC group was higher than that from shRNA‐Trop2 group (*P* < 0.05; Figure 4C).

**Figure 4:** Trop2 depletion inhibits metastasis of GC cell line in vivo*. *A, The lung from PBS control (n = 5), shRNA‐NC‐BGC823 (n = 5), and shRNA‐Trop2‐BGC823 group (n = 5). B, is the statistic graph of A, columns, mean lung weight (g); Bars, ±SD, *means compared with shRNA‐NC group, *P* < 0.05, **means compared with PBS group, *P* < 0.001, *t* test. C, The representative picture of lung from shRNA‐NC and shRNA‐Trop2 group. The weight of lung harboring metastases was evaluated between control and Trop2 depletion group. D, representatives of hematoxylin staining in lung tissue derived from PBS, shRNA‐NC‐BGC823, and shRNA‐Trop2‐BGC823 injected mice. Ki67, Trop2, and vimentin staining in lung tissue derived from PBS, shRNA‐NC‐BGC823, and shRNA‐Trop2‐BGC823 injected mice

Then, we further detected the Trop2, vimentin, and ki67 expression in lungs by immunostaining (IHC) analysis. As shown in Figure 4D, the level of Trop2 and vimentin expression in lungs from the shRNA‐NC group was much higher than those from shRAN‐Trop2. In comparison with that in shRNA‐NC group, the positive rate of ki67 expression was significantly decreased in shRNA‐Trop2 and PBS control group. These results indicated that Trop2 might induce EMT and prompt metastasis in vivo.

### 3.4 High expression Trop2 and vimentin positively associated with metastasis in human gastric cancer

Finally, we used IHC analysis to determine whether the expression level of the EMT marker vimentin could have a correlation with that found in the Trop2 in clinical samples. In a previous study, we already found Trop2 expression to be higher in GC tissues than in gastric cancer neighbor tissues by IHC, and that Trop2 is a useful prognostic biomarker for GC^25^. Therefore, in our present study, gastric cancer neighbor tissues (GCN), nonmetastatic gastric cancer (NMGC) tissues, and metastatic gastric cancer tissues (MGC) were collected from patients with gastric cancer. Trop2 and vimentin protein expression was determined in 248 cases of primary GC tissues and 86 cases of matched adjacent tissue by IHC (Table 1). We observed that highly expressed vimentin was consistent with the high expression of the Trop2 in GC tissues (Table 2), especially in MGC tissues (Figure 5). Furthermore, we found that high Trop2 and high vimentin expression in GC was associated with differentiation, TNM stage, distant metastases (Tables 3 and 4). GC patients with vimentin+ or Trop2+/vimentin+ expression also had poor OS rates (Figure 5B1‐B2).

**Table 1:** vimentin and Trop2 expression in gastric tissues

Characteristics	n	Vimentin expression		Pearson *x* ^2^	*P*	Trop2+/vimentin+	Pearson *x* ^2^	*P*
		Low or no	High					
Stomach								
Cancer	248	50 (20.16)	198 (79.84)	14.246	0.014*	142 (83.52)	35.867	0.002*
Matched adjacent tissue	86	28 (32.56)	58 (67.44)			29 (17.06)		

*x* ^2^ and *P* values for stomach overall include all types gastric tissues.

* *P *< 0.05.

**Table 2:** Association between expression of Trop2 and vimentin in gastric cancer

Vimentin expression (%)	n	Trop2 expression (%)		Pearson *x* ^2^	*P*
		Low or no	High		
Low or no	80	31 (62.00)	19 (38.00)	19.927	**<0.001** *
High	198	56 (28.28)	142 (71.71)		

* *P *< 0.05.

Bold values are statistically significant.

**Figure 5:** The expression level of Trop2 and vimentin was positively correlated in GC patients. A, The expression of Trop2 and vimentin was detected in 248 cases of GC patient tissues by IHC. a1‐2, low or no expression of Trop2 in GCN samples (IHC score, 30). b1‐2, high expression of Trop2 in NMGC samples (IHC score, 180).c1‐2, high expression of Trop2 in MGC samples (IHC score, 230). a3‐4, low or no expression of vimentin in GCN samples (IHC score, 100). b3‐4, high expression of vimentin in NMGC samples (IHC score, 150).c3‐4, high expression of vimentin in MGC samples (IHC score, 250). B, Survival curves for gastric cancer using the Kaplan‐Meier method and the log‐rank test. B1, Overall survival curves for patients with low or no expression of vimentin (blue line, 1), high expression of vimentin (green line, 2). B2, Overall survival curves for patients with Trop2−/vimentin−expression (blue line, 1), Trop2+/vimentin− (green line, 2), Trop2−/vimentin+ (gray line, 3), and Trop2+/AREG+ (purple line, 4)

**Table 3:** Association of high expression of Trop2+/vimentin+ with clinicopathologic characteristics in GC patients

Characteristics	n	Vimentin expression (%)		Pearson *x* ^2^	*P*	Trop2+/vimentin+	Pearson *x* ^2^	*P*
		Low or no	High					
Total	248					**141** (**56.85)**		
Gender								
Male	182	37 (20.33)	145 (79.67)	**0.012** *	0.913	101 (40.73)	2.110	0.550
Female	66	13 (19.70)	53 (80.30)			40 (16.13)		
Age								
<60	103	20 (19.42)	83 (80.58)	0.061	0.806	58 (23.39)	4.526	0.210
≥60	145	30 (20.69)	115 (79.31)			84 (33.87)		
Histological type								
Tubular	216	43 (19.91)	173 (80.09)	3.783	0.286	122 (49.19)	6.900	0.648
Mucinous	17	3 (17.65)	14 (82.35)			11 (4.44)		
Signet ring cell	10	4 (40.00)	6 (60.00)			5 (2.02)		
Others^a^	5	0 (0.00)	5 (100.00)			3 (1.21)		
Differentiation								
Well	23	7 (30.43)	16 (69.57)	2.884	0.236	9 (3.63)	12.759	**0.047** *
Moderate	57	8 (14.04)	49 (85.96)			41 (16.53)		
Poor	168	35 (20.83)	133 (79.17)			91 (36.69)		
TNM stage								
0	13	6 (46.15)	7 (53.85)	7.258	**0.027** *	3 (1.21)	15.503	**0.017** *
I + II	135	29 (21.48)	106 (78.52)			71 (28.63)		
III + IV	100	15 (15.00)	85 (85.00)			67 (27.02)		
Tumor size								
T0	58	15 (25.86)	43 (74.14)	1.535	0.464	28 (10.08)	8.616	0.196
T1a + T1b + T2	39	7 (17.95)	32 (82.05)			21 (8.47)		
T3 + T4a + T4b	151	28 (18.54)	123 (81.46)			92 (37.10)		
Distant metastases								
M0	88	40 (45.45)	48 (54.55)	54.212	**<0.001** *	32 (12.90)	52.369	**<0.001** *
M1	160	10 (6.25)	150 (93.75)			109 (43.95)		

a others include pallipary adenocarcinoma, 3 cases; adeno‐squamous carcinoma, 2 cases; and neuroendocrine carcinoma, 1 case.

* *P *< 0.05.

Bold values are statistically significant.

**Table 4:** Univariate and multivariate analysis of prognostic markers for overall survival in gastric cancer

	Univariate analysis			Multivariate analysis		
	HR	*P *> |*z*|	95% CI	HR	*P *> |*z*|	95% CI
Vimentin expression						
High vs Low or no	2.167	**0.017** *	1.151‐4.079	—	—	—
Trop2+/vimentin+ vs Trop2−/vimentin−	1.603	**<0.001** *	1.272‐2.019	1.544	**0.007** *	1.125‐2.119
Age						
<60 vs ≥60	0.629	0.074	0.378‐1.947	—	—	—
Gender						
Male vs Female	1.238	0.463	0.700‐2.191	—	—	—
Histological type						
Tubular vs Mucinous vs signet ring cells vs others^a^	0.776	0.233	0.511‐1.178	—	—	—
Differentiation						
Well vs Moderate vs Poor	2.244	**<0.001** *	1.481‐3.400	—	—	—
TNM stage						
0 vs Ia + Ib vs IIa + IIb vs IIIa + IIIb vs IIIc + IV	6.949	**<0.001** *	3.931‐12.285	5.731	**<0.001** *	3.143‐10.452
Tumor size						
T0 vs T1a + T1b + T2 vs T3 + T4a + T4b	2.387	**<0.001** *	1.721‐3.310	—	—	—
Distant metastases						
M0 vs M1	2.297	**0.002** *	1.351‐3.905	—	—	—

a Others include pallipary adenocarcinoma, 3 cases; adeno‐squamous carcinoma, 2 cases; and neuroendocrine carcinoma, 1 case.

* *P* < 0.05.

Bold values are statistically significant.

## 4 DISCUSSION

China has more GC patients than any other country and due to high rate of migration, invasion, and drug‐resistance, and currently, patients in an advanced stage of the GC have a poor survival rate.^27^, ^28^ Epithelial‐mesenchymal transition (EMT) is a phenomenon in which epithelial cells change into mesenchymal cells in both normal or pathological conditions and more, and more research indicates that the EMT phenomenon has an important role in the transition from early to invasive carcinomas.^29^, ^30^ Multilayer cellular structures’ normal epithelial organization is not conductive to the migration and invasion of malignant tumor cells.^31^, ^32^ So, through the EMT phenomenon, tumor cells lose epithelial phenotype but obtain a mesenchymal phenotype.^33^ In our present study, we found that Trop2 was able to induce the EMT phenomenon in gastric cancer cell lines. It has been previously shown that Trop2 drives hyperplasia and stem cell self‐renewal through beta‐catenin signaling pathway,^34^ and this opinion concurs with the findings of this study.

It also be reported that Trop2 is not up‐expressed in the lung adenocarcinoma^12^; furthermore, Wang et al^17^ also reported that loss of Trop2 in squamous cell carcinoma fail to inhibit keratinocyte transformation, which lead to keratinocytes to pass through EMT and tumor formation. The research that both gain and loss of Trop2 function stimulate strong phenotypes indicated that this protein possesses a pleiotropic mechanism of action and potent signaling activities.

As one of the core factors of the Wnt signal pathway, β‐catenin widely exists in all kinds of cells and has multiple functions.^35^, ^36^ β‐catenin mainly exists in the membrane of cells and to a lesser extent in the cytoplasm of cells. Its main function being the regulation of intercellular adhesion and is also involved in the expression of genes.^37^ The level of expression of β‐catenin also directly impacts the activation of the Wnt signal pathway.^38^ When the degradation of β‐catenin becomes an obstacle, too much β‐catenin accumulates in the endonuclear membrane leading to cancer via an abnormal activation of the Wnt signal pathway.^39^ In 2012, Tanya et al reported that the function of Trop2 requires the presence of β‐catenin in nucleus. Overexpression of Trop2 induced cyclin D1 and c‐myc expression, which is the downstream target of β‐catenin. Furthermore, they demonstrated that Trop2 could drive cell sphere formation and hyperplasia only in the presence of β‐catenin in vitro and in vivo.^34^ Gene ontology analysis reported that Trop2 impacts Wnt/β‐catenin, TGF‐β, and phosphoinositide 3‐kinase (PI3K) pathways; all have important functions in tumorigenesis.^40^, ^41^, ^42^ In our study, we investigated whether Trop2 could upregulate the expression of the mesenchymal phenotypic (vimentin and fibronectin) and downregulate the epithelial phenotypic (E‐cadherin) and we also investigated whether Trop2 is involved in β‐catenin/TGF‐β1‐mediated EMT. Trop2 and EMT regulators β‐catenin were also involved in the overexpression in EMT model cell lines. Trop2 is physically associated with β‐catenin to induce EMT phenomenon by co‐immunoprecipitation. Trop2 knockdown reduces the protein expression of the vimentin and β‐catenin. Moreover, OE‐Trop2 induces the nuclear accumulation of β‐catenin; meanwhile, TGF‐β1 mediates the nuclear accumulation of β‐catenin, which is also diminished by Trop2 inhibition.

The above results indicate that Trop2 is involved in β‐catenin/TGF‐β1‐mediated EMT in GC. Collectively, our results indicate intricate mechanisms, in which Trop2 regulates the transcription of β‐catenin target genes and EMT, while Trop2 facilitates the transcription of β‐catenin target gene, but moreover promotes the nuclear translocation and accumulation of β‐catenin, thereby increasing its transcription activity.

As is known, EMT endows cells with the properties of being migratory and invasive and accelerates stem cell properties, promotes immunosuppression and deters apoptosis and senescence.^43^, ^44^ Thus, the mesenchymal program is associated with the capacity of cells that can migrate to distant organs and initiate metastasis.^45^ There have been reports that β‐catenin nuclear accumulation is a hallmark of β‐catenin transcriptional activation.^23^, ^46^ However, it is still unclear how Trop2 regulates the nuclear translocation of β‐catenin and the detailed regulatory mechanism needs to be further researched.

In our studies, we also found snail overexpression (apart from Trop2 and β‐catenin) in the TGF‐β1‐induced EMT model cell lines. Therefore, it is likely that other signal pathways maybe involved in Trop2 in association with the β‐catenin regulation EMT mechanism. It was also reported that snail promotes Wnt target gene expression and interacts with β‐catenin, so we speculate that snail perhaps has a similar role in the EMT program, but in order to elucidate the mechanism, further study is needed. Furthermore, we also found vimentin highly expressed in GC tissues, compared with that of the gastric cancer neighbor tissues, which is in accordance with viewpoint of the Ruixia Xie et al.^47^ Trop2+/vimentin+ co‐expression was associated with poor prognosis and may be regarded as useful prognostic biomarker in GC.

Recent evidence suggests Trop2 is a regulator of self‐renewal, proliferation, and transformation. However, the molecular mechanism of Trop2 in tumor metastasis and progression is still unclear. In this study, we show that Trop2 positively promotes EMT phenomenon through binding to β‐catenin, thereby forming a positive feedback loop for to amplify the EMT phenomenon.

## CONFLICT OF INTEREST

The authors have declared that no competing financial interests exist.
